# The protective effect of Pentoxifylline on testopathy in male rats following Dimethyl Nitrosamine administration: An experimental study

**DOI:** 10.18502/ijrm.v17i10.5292

**Published:** 2019-11-07

**Authors:** Mohammad Reza Salahshoor, Azita Faramarzi, Shiva Roshankhah, Cyrus Jalili

**Affiliations:** ^1^Department of Anatomical Sciences, Medical School, Kermanshah University of Medical Sciences, Kermanshah, Iran.; ^2^Fertility and Infertility Research Center, Health Technology Institute, Kermanshah University of Medical Sciences, Kermanshah, Iran.

**Keywords:** Dimethyl nitrosamine, Reproductive, Pentoxifylline, Rat.

## Abstract

**Background:**

Nitrosamines as a carcinogenic agent has unfavorable effects on some of the male reproductive parameters. Pentoxifylline (PX) is a xanthine derivative used as a drug inhibiting the inflammatory factors, reducing blood viscosity, improving peripheral blood flow, and so on. **Objective:** The aim of the present study is to evaluate the effects of PX against Dimethyl nitrosamine (DMN)-inducing the damage to the reproductive parameter of male rats.

**Materials and Methods:**

In this experimental study, 48 male Wistar rats (8 wk, 220-250 gr) were randomly assigned to eight groups (n = 6/each): normal control and DMN control groups (40 mg/kg); PX groups (25, 50, 100 mg/kg), and DMN + PX groups (25, 50, 100 mg/kg). Treatments were administered intraperitoneally and the gavage applied daily for 28 days. The sperm parameters, spermatogenesis index, total antioxidant capacity, testosterone level, and seminiferous tube diameter were assessed.

**Results:**

The values of all parameters reduced significantly in the DMN control group compared to the normal control group (p < 0.001). The PX and PX + DMN treatments at all entirely doses improved all parameters significantly compared to the DMN control group (p < 0.001).

**Conclusion:**

DMN caused detrimental effects on reproductive parameters. Also, no significant modifications were observed in PX treatments at all doses compared to the normal control group. PX compensated the toxic effect of DMN on reproductive parameters.

## 1. Introduction

Male infertility is a complex disorder affecting a large part of the community population. Disruption of any stage in the sequence of fertility causes definite failure in this process (1). Free radicals, by attacking unsaturated fatty acids and alkylation of protein groups and other cellular macromolecules, resulting in lipid peroxidation in the cell membrane, change in the enzyme activity, and finally leading to cellular damage and necrosis (2). The production of reactive oxygen species (ROS) result in break in the cell cycle and induce the apoptosis process, thereby reducing the daily sperm production as well as the total number of sperms (3). Nitrosamines are the products of the reaction among nitrite, free amino acids, and amines (4). The human exposure to nitrosamines is carried out through a variety of routes, especially food, including meat. They are extensively found in foods and natural products, artificial substances, chemicals, cigarettes, detergents, anti-stains, solvents, medicines, leather and plastics products, as well as cosmetics (5). The human contact with DMN compounds is associated with the risk of esophageal, gastric, and bladder cancers (6). Nitrosamines by the ability of diazonium ions formation have the potential to induce DNA damage. These compounds also apply activation of cytochrome P-450 enzyme by the formation of diazonium and oxonium ions as well as alpha-hydroxylation metabolites (7). Nitrosamines induce oxidative stress and produce free radicals in the body resulting in cellular damage (8). However, the cell defense system of the body is not fully capable for damage prevention of free radicals, especially under acute conditions, the use of antioxidant agents helps reducing damage and preventing the disease caused by it (9). Pentoxifylline (PX) as one of methyl xanthine derivatives and noncompetitive inhibitors of phosphodiesterases increases the intracellular adenosine monophosphate (cAMP) which activates protein kinase and inhibits tumor necrosis factor, thereby reducing the leukotriene production and inflammation, and enhances the innate immunity (10). PX also has antioxidant effects which seem to be performed by activating neutrophils in response to superoxide produced by NADPH oxidase (11). In addition, the use of PX powder can increase sperm motility (12). So, the purpose of the present study was to assess the protective effect of PX on reproductive dysfunction of male rats induced by the administration of Dimethyl Nitrosamine (DMN). To the best of our knowledge, this preliminary study is the first investigation to access the protective effect of PX on reproductive parameters of male rats induced by DMN.

## 2. Materials and Methods 

### Animals

In this experimental study, 48 male Wistar rats (weighing 220-250 gr, 8 wk) purchased from the Pasteur Institute and housed in the animal home of medical school. During the present study, the animals were kept under standard conditions of 12 hr light/dark cycle and 22 ± 2°C in special cages and on a straw bed. Water and food were freely available to the animals. The animals were fed standard food and treated municipal drinking water.

### Study groups and treatment of animals

Forty-eight male rats were randomly divided into eight groups with six rats in each group. In the first group, the normal control group, each rat received normal saline (by oral gavage and injection) equivalent to the number of experimental groups. In the second group, the control group of DMN, each animal received a single dose of 40 mg/kg DMN intraperitoneally with normal saline as a solvent of DMN. Each animal in the third, fourth, and fifth groups, the PX administration groups, received 25, 50, and 100 mg/kg, of PX orally (gavage), respectively, at 10 am for 28 days. In the sixth, seventh, and eighth groups, DMN + PX administration groups, each animal received a single dose of 40 mg/kg DMN in order to induce reproductive parameters damage, and then received 25, 50, and 100 mg/kg of PX oral gavage, respectively, at 10 am for 28 days.

### Animal dissection and sampling

Twenty eight days after the treatment of animals and free access to water and food, the rats belonging to each group were euthanized regularly and sequentially by the vapor of ether-impregnated cotton (Merck Co., Germany).

The blood samples were collected from the heart without thoracotomy. The blood was poured into test tubes, kept in a 37°C incubator for 20 min and centrifuged at 255 ×g for 15 min. The blood serum was isolated and part of it was kept at -70°C for measuring the total antioxidant capacity, nitric oxide, and testosterone levels. Then, the chest and abdomen of the animals were cut respectively. The tail of epididymis was isolated from the testes and placed in DMEMF12/FBS5% culture medium. The testicles were removed from the abdominal cavity and fixed in a 10% formalin solution.

### Sperm cells collection 

The epididymis caudal part was cut and used for sperm parameters evaluation. The caudae of epididymides were crushed and placed in warmed petri dish containing 10 ml Hams F 10 at 37°C. The sperm were dispersed into Hams F 10. After 15 min, 10 µl of mixed suspension was observed by a light microscope at 400× magnification. The left testis was used for histological staining.

### Sperm viability

In this method, eosin stain was used to identify living sperm cells from dead ones based on the transmission of stain through the cell membrane of dead cells and repelling from the cell membrane of living cells. At the end of the given time, about 20 μl of the medium containing semen fluid was collected from each petri dish, and mixed with an equal volume of eosin stain solution (about 20 μl). After 2-5 min, a part of the mixture was poured onto a neobar culture slide. The living and dead sperm cells lack stain and become pink subsequently. The prepared culture slide was examined with 40× magnification. At least 100 sperm cells were calculated from each random sample according to the 10 fields of imagining, and the percentage of living sperm cell was documented.

### Sperm progressive motility 

Four degrees of sperm motility was calculated according to the WHO guidelines (2010) (13), class A: progressive motility. Progressive motility of the sperm cells of each sample was examined by an optical microscope with 40× magnification in 10 fields of view. For this purpose, about 50 μl of semen liquid culture medium was taken first and then placed on a culture slide that was previously cleaned and dried with alcohol and finally examined by the microscope. Sperm cell counting was performed through a cell count device, and about 100 sperm cells were counted in each sample. In all experimental and control groups, the counting was repeated.

### Sperm count 

To analyze the number of sperm cells, 400 μl of the sperm suspension was diluted with formaldehyde fixative (Sigma; USA). Approximately, 15 μl was transferred from the diluted solution into a hemocytometer by a Pasteur pipette. The hemocytometer was located into a petri dish with dampened filter paper and allowed to stand for 10 min. The stable sperms were counted and assessed per 250 small squares of the hemocytometer using a ×40 objective. The number of sperm per mm${}^{3}$ was calculated using the formula: the number of sperm counted × the dilution/number counted in mm${}^{2}$ × the depth of the chamber.

### Sperm cells morphology 

Sperm smears from every case were used for sperm morphology evaluation. Eosin/nigrosin staining was done to assess normal morphology. 10 µl of eosin dye was added to 10 µl of sperm suspension and mixed gently. Then, the slides were seen using light microscope at 400× magnification. 400 sperm were assessed on the slide.

### Seminiferous tubules 

After the fixation of testes, they were dehydrated, cleared, and embedded. Sections of 5 μm in thickness were prepared and hematoxylin and eosin staining were applied. More than 30 segments were organized from each block. The seminiferous tubules were measured using a Motic camera and software (Moticam 2000; Spain). The mean diameter of the seminiferous tubules was determined for each testis.

### The ferric reducing ability of plasma (FRAP) method

The ferric reducing ability of plasma (FRAP) procedure was done to evaluate the serum total antioxidant capacity. In this method, the plasma ability to balance the ferric ions was evaluated. This procedure needs a great volume of Fe${}^{\mathrm{III}}$. When the Fe${}^{\mathrm{III}}$-TPTZ in acidic pH reversed to Fe${}^{\mathrm{II}}$, blue dye was formed. The absorption was performed at the wavelength of 600 nm. The defining factor of the Fe${}^{\mathrm{II}}$-TPTZ speed and blue dye were the main power of the sample. The total antioxidant capacity quantities were strategized by the standard curve, as well as different concentrations of iron sulfate.

### Testosterone

The collected blood sample was centrifuged to get the serum for 15 min with 5,000 gr at 23°C. Subsequently, the serum samples were kept in a deep freezer (-18°C). The serum testosterone level was examined through the ELISA (Abcam 108666, USA) technique.

### Spermatogenesis index

Seminiferous tubules were assessed for spermatogenesis index (SI) by Johnson's score. Based on it, a grading system from 10 to 1 was given to each of section of Seminiferous tubule ranging from complete to no cells spermatogenesis(14) (Johnsen, 1973).

### Ethical consideration

All investigations conformed to the ethical and humane principles of research and were approved by the Ethics Committee of our institute (Kermanshah University of Medical Sciences Committee on the Use and Care of Animals, IR.KUMS.REC.1396.21).

### Statistical analysis

After extracting the information, the Kolmogorov-Smirnov test was first conducted to confirm data compliance of the normal distribution. One way analysis of variance (one-way ANOVA) was used for statistical analysis and the Tukey post-hoc test was used to determine the difference between the groups. The Statistical Package for the Social Sciences version 16 (SPSS Inc., Chicago, IL) was used for data analysis, the results were expressed as mean ± standard error, and p < 0.05 was considered significant.

## 3. Results

### Sperm viability, progressive motility, count, and normal morphology

DMN caused a significant reduction in viability, progressive motility, count, and normal morphology compared to the normal control group p < 0.001). No significant variations were detected in PX groups compared to the normal control group (p = 0.19, p = 0.11, p= 0.24, p= 0.31). Also, the mentioned parameters in all PX and DMN + PX groups increased significantly compared to the DMN control group p < 0.001) (Figure 1).

### Seminiferous tubules 

DMN induced a considerable decrease in the diameter of seminiferous tubules compared to normal control group (p < 0.001). No significant

change was seen in PX groups compared to the normal control group (p = 0.14). Seminiferous tubule diameter in all PX and DMN + PX groups enhanced significantly compared to the DMN control group (p < 0.001) (Figures 2 and 3).

### Total antioxidant capacity 

The serum total antioxidant capacity was significantly decreased in DMN control group compared to the normal control group (p < 0.001). The serum total antioxidant capacity was considerably increased in PX groups compared to DMN control groups (p < 0.001). Also, it improved considerably in DMN + PX groups compared to the DMN control group (p < 0.001) (Figure 4).

### Testosterone

DMN caused a significant decrease in the testosterone hormone level compared to the normal control group (p < 0.001). No significant alterations were detected in PX groups compared to the normal control group (p = 0.23). Furthermore, the testosterone hormone level in all PX and DMN + PX groups improved significantly compared to the DMN control group (p < 0.001) (Figure 5).

### Spermatogenesis index

DMN caused a significant decrease in the spermatogenic index compared to the normal control group (p < 0.001). No significant changes were observed in all PX groups compared to the normal control group (p = 0.12). Moreover, spermatogenic index in all PX and DMN + PX groups showed a significant increase compared to the DMN control group (p < 0.001) (Figure 6).

**Figure 1:** Effect of DMN, PX, and PX + DMN on sperm parameters. Comparison of sperm viability (A), progressive motility (B), count (C), and normal morphology (D) among treatment groups. *Significant decrease in the DMN control group compared to the normal control group (p < 0.001). †Significant increase in all PX groups compared to the DMN control group (p < 0.001). ‡Significant increase in all PX + DMN groups compared to the DMN control group (p < 0.001).

**Figure 2:** Comparison of seminiferous tubule diameter in treatment groups. *Significant decrease in the DMN control group compared to the normal control group (p < 0.001). †Significant in all PX groups compared to the DMN control group (p < 0.001). ‡Significant in all PX + DMN groups compared to the DMN control group (p < 0.001).

**Figure 3:** Effect of Nitrosamine, PX, and PX + DMN on the germinal layer of seminiferous tubules (magnification ×40). The structure of normal seminiferous tubule was observed in the control group (A) and PX group (B). A decrease in thickness of the germinal layer and sperm cells inside the seminiferous tubules was observed in the DMN control group (C). The structure of normal seminiferous tubule was observed in PX + DMN group (D). The black arrow indicates germinal layer (reduction in epithelial height and irregularities in the structure of the margin of tubules), the yellow arrow indicates structural destruction of the membrane seminiferous tubules, and the blue arrows indicate sperm cells.

**Figure 4:** Comparison of total antioxidant capacity in treatment groups. *Significant decrease in the DMN control group compared to the normal control group (p < 0.001). †Significant increase in all PX groups compared to the DMN control group (p < 0.001). ‡Significant increase in all PX + DMN groups compared to the DMN control group (p < 0.001).

**Figure 5:** Comparison of testosterone hormone level in treatment groups. *Significant decrease in the Nitro DMN control group compared to the normal control group (p < 0.001). †Significant increase in all PX groups compared to the DMN control group (p < 0.001). ‡Significant increase in all PX + DMN groups compared to the DMN control group (p < 0.001).

**Figure 6:** Comparison of spermatogenesis index in treatment groups. *Significant decrease in the DMN control group compared to the normal control group (p < 0.001). †Significant increase in all PX groups compared to the DMN control group (p < 0.001). ‡Significant increase in all PX + DMN groups compared to the DMN control group (p < 0.001).

## 4. Discussion

The present study showed that viability, motility, count, and normal morphology of sperm cells in the DMN control group reduced significantly compared to the normal control group. Also, this material decreased the level of total serum antioxidant capacity. DMN induced oxidative stress in testicular tissue which is proved by the enhancement in the levels of ROS and lipid peroxidation and a decrement in antioxidant enzymes activity similar total antioxidant capacity. The quantity of antioxidant of testis can be detrimental by high levels of unsaturated fatty acids of related cell membrane and cell proliferation as well as high metabolism (15).

Sadik *and colleague showed* that the DMN-induced hepatocarcinogenesis of male rats significantly reduces the serum levels of total antioxidant capacity, which confirms the results of the present study (16).

It seems that ROS affects the synthesis of DNA and RNA in sperms and inhibits the function of mitochondria (17). It is possible that oxidative stress conditions also act in the same way on sexual germ cells and disrupt their divisions and differentiation so that the number of spermatogonia affected on the basement membrane reduced as well as the number of primary and secondary spermatocytes, spermatids, and adult sperms (18). Meanwhile, oxidative stress can disrupt the spermatogenesis process resulting in the formation of defective gametes with remodeled chromatin that is susceptible to be attacked by the free radicals leading the reduction of the number of spermatogonia, spermatocytes, spermatids, and spermatozoa (19). In agreement with the present study, Khan *and others* showed that arsenic-induced oxidative stress in male rats caused ROS production, deformity of sperm, and a significant reduction in the motility and number of sperms and testosterone levels in comparison to the control group (20). The first consequence of ROS attack to membrane structures of cells is the occurrence of peroxidation within the cell membrane and organelles. Since the sperms during the stages of spermatogenesis lose a large amount of their cytoplasm (lack of antioxidant systems), it seems to be more sensitive to increase the accumulation of ROS in the environment than somatic cells (21). It seems that high levels of ROS can reduce spermatozoal motility due to the effect on Ca${}^{++}$ channels and reduction of spermatozoal ATP reserves (22). Also, the reduction in glutathione levels can reduce spermatozoal motility (23). It seems that the plasma membrane of sperms is susceptible to oxidative damage due to the presence of large amounts of unsaturated fatty acids leading to reduced motility and viability of sperms (24). Khan *and coworkers* showed that arsenic-induced oxidative stress in male rats induced ROS production, sperm deformity, DNA degradation, reduced fertility index, motility, and number of sperm and level of testosterone in comparison with the control group (20). Although, it was shown that the administration of DMN in male rats caused a significant reduction in the number of sperm motility and survival status of sperm cells compared to the control group, which confirms the results of the present study (25).

In addition, the present study showed that PX and DMN + PX administration significantly increased the viability, motility, count, and normal morphology of sperm cells compared to the DMN control group. PX is a methyl xanthine derivative enhancing the sperm motility by increasing the intracellular calcium concentration and membrane penetration of cAMP analogs that inhibit the action of phosphodiesterase (26). According to the low amount of cytoplasmic enzymes, no potential is found for the regeneration of oxidative damage, and antioxidants and antioxidant enzymes are crucial for the semen fluid to protect against oxidative damage (9). PX has anti-inflammatory properties, which seems to reduce the level of LPO and prevent cells damage (27). It was shown that the proximity of sperm with PX induced motility in immotile sperms (28). Also, in line with our study, Nabi *and colleague*. found that in-vitro application of PX eliminates detrimental effect of cryopreservation on sperm motility without ultrastructure alterations (29).

However, we found that the serum level of total antioxidant capacity improved significantly in the PX and PX + DMN groups compared to the DMN control group. In this study, the reduction in the level of total antioxidant capacity shows the effects of oxidative stress regarding the DMN on reproductive parameters. In the present study, the improved levels of total antioxidant capacity treated with PX highlight the antioxidant and anti-lipid peroxidation effects of PX.

The present study showed that the diameter of seminiferous tubules and testosterone levels in the DMN control group reduced significantly compared to the normal control group. In the PX and DMN + PX groups, a significant increment was observed in the normal morphology of sperm cells, the diameter of the seminiferous tubules, and the testosterone level compared to the DMN control group. DMN can induce oxidative stress activity, DNA damage, lipid peroxidation, as well as the formation of additional protein compounds by producing ROS such as superoxide and hydrogen peroxide (30). It seems that septal cells of seminiferous tubules rapidly differentiated in the DMN control group and released from the septum of tubules, which increased the diameter of the tubules (31). In addition, increasing ROS with increasing lipid peroxidation leads to induction of tubules atrophy and apoptosis of the germ cells (32). It seems that a significant relationship is found between the production of oxygen species in sperms and disturbed morphology of sperms. The conditions for increasing the number of free radicals including the destruction of cells of enveloping tissue, damage to Sertoli cells, the collapse of cytoplasmic bridges, and, consequently, a reduction in the number of sperms and an increase in sperms' motility (33). The administration of DMN can lead to a significant reduction in testosterone levels due to oxidative stress (25). The study of Dutra *et al*. consistent with the present study showed that the administration of PX significantly increased the diameter of seminiferous tubules and testosterone level (34). It seems that, along with antioxidant properties of PX, the vasodilatation and the increased blood supply are the factors causing the enhancement of production of testosterone in this study (35). However, the present study showed that DMN decreases the SI. Also, all PX and PX + DMN groups increase SI compared to the DMN control group, significantly. The SI changed from level 8 (few sperm) to 5.5 (no sperm and many spermatocytes) during the administration of DMN. Although, PX treatment was increased SI.

## 5. Conclusion

A limitation of this study was the lack of information on the exact mechanism about the action of protective effects of PX. Therefore, future studies are needed.

Our finding demonstrated that DMN can produce pathological changes in testicular tissue and abnormality in sperm parameters. In addition, PX is able to ameliorate the detrimental effects of DMN.

##  Conflict of Interest

The authors declare that they have no conflict of interest.
